The article "Evaluation of Time Consumption for Debonding Brackets Using Different Techniques: A Hospital-Based Study" was published in 2021. Journal: J Healthc Eng.

# Evaluation of Time Consumption for Debonding Brackets Using Different Techniques: A Hospital-Based Study

**DOI:** 10.1155/2021/5567863

**Published:** 2021-08-24

**Authors:** Neelutpal Bora, Putul Mahanta, Ranjumoni Konwar, Bharati Basumatari, Chiranjita Phukan, Deepjyoti Kalita, Senjam Gojendra Singh, Sangeeta Deka

**Affiliations:** ^1^Dentistry, Assam Medical College and Hospital, Dibrugarh 786002, Assam, India; ^2^Forensic Medicine and Toxicology, Assam Medical College and Hospital, Dibrugarh 786002, Assam, India; ^3^Radiology, Fakhruddin Ali Ahmed Medical College and Hospital (FAAMC), Barpeta, Assam, India; ^4^Medicine, Tezpur Medical College and Hospital, Tezpur, Assam, India; ^5^Microbiology, All India Institute of Medical Sciences, Rishikesh, Uttarakhand, India; ^6^Department of Psychiatry, Regional Institute of Medical Sciences, Imphal, India

## Abstract

**Materials and Methods:**

A total of 80 human premolars were included in this study. The samples were first arranged following a standard protocol for bracketing and then debonded using the ultrasonic scaler (US), debonding plier (DP), ligature cutter (LC), and thermal method (TM). Depending on the technique applied for debonding, the specimens were randomly divided into four groups with 20 samples, each keeping a 1 : 1 ratio. During the debonding process, the time taken for each bracket removal was recorded using a stopwatch. To assess the difference in mean time required for debonding among the four techniques, one-way ANOVA test was applied along with Tukey's HSD to compare the two methods.

**Results:**

The time range and the mean time required for the four techniques analyzed show that the DP method has the highest range of time needed for debonding with 0.97–2.56 seconds, while LC methods have the least time range taking 0.46 to 1.79 seconds. TM's mean time to debond is the highest at 1.5880 seconds. LC method has the lowest mean debonding time of 0.9880 seconds. The one-way ANOVA test has shown the mean debonding time required by the four techniques to be significantly different (*p* < 0.001). Tukey's HSD multiple comparisons also show that the mean time to debond using the LC method is substantially less than the other three methods (*p* < 0.001).

**Conclusion:**

The mean debonding time for the TM was substantially the highest, followed by the US and DP. Debonding with the LC technique required the least time. This study shows some limelight towards the effectiveness of the LC method as it is the least time-consuming technique.

## 1. Introduction

The debonding process removes brackets with all remaining left-out adhesives from the enamel surface [1]. To restore the enamel surface, orthodontists are on the hunt for an effective and time-economic debonding method. Many have addressed the volume of enamel loss and time consumption for the bracket removal process [2–4], yet to find out the best time-economic technique of the debonding process.

The typical features of a standard orthodontic application consist of esthetical look, minimal enamel damages, and less time consumption. The dental surgeon needs to provide their patients with the appliances which have all these characters. The demand for orthodontic care has risen from 14% to 27% in recent times [5] and is thought to increase in the coming years [6].

Thus, like that of other branches, an effort for evaluating simplified and comfortable techniques of debonding from the patient perspective is made on [7]. Numerous orthodontists use their approach to debond the brackets on a trial basis, lacking the information of damage caused to the bracketing areas [8], including the time consumption. Hence, no agreement has reached the best bracket removal practice [9, 10], although the less time-consuming method was mentioned in a review [11].

Feldspar, or alumina, was merged with the first crown during the early period of the 20^th^ century. Leucite was then put into feldspar because of the significant discrepancies in the thermal increase of the overlying ceramic and the underlying metal alloy in the 1960s [12]. As the ceramic brackets have a notable failure rate [13], they demanded a furtherimproved method. Further ceramic bonding needs a particular etching protocol as it shows resistance to acids [14] relatively. The same research reveals the type of conditioning agent as the main factor for evaluating the bond intensity. Hence, in orthodontic practice, only the most effective method is used.

The main content of the ceramic brackets is aluminium oxide (alumina). Depending on the production procedures, the two types of ceramic brackets are used: monocrystalline and polycrystalline [15].

Aluminium oxide was first melted and then allowed to cool gradually to form the crystal to make the monocrystalline brackets. The impurities and imperfections are minimal here without the addition of the binding materials. During the process of crystallization, it is shaped like a bracket [16].

The polycrystalline brackets are produced by sintering the fragments of aluminium oxide together. The components are intermingled along with the binding material, shaped to a bracket. The shaped bracket is then fired to burn the binder, and the aluminium oxide fragments then fuse, which is an economical procedure [16].

The metal brackets have more fracture toughness in comparison to ceramic brackets. The ceramic brackets are shattered more during the time of bracket removal [17]. The process of ceramic bracket removal produces lots of inconveniences even though exceptional aesthetically. It may be associated with tie wing failure, enamel fracture, pain, and irritation during the process of bracket removal [18, 19]. Thus, the time required for debonding may be varied. The fracture of the enamel at the time of bracket removal creates a great concern aesthetically. Furthermore, more time is needed for bracket tie wing failure for debonding by grinding with a diamond bur [20].

Still, ceramic brackets have an excellent reputation, which were introduced in the mid-1989 [21], due to their biocompatibility, attractive gazes, and best biomechanical nature in restorative dental practices [12, 22]. Yet, the metallic brackets are still considered as the gold standard as a bonding method [23].

The ceramic brackets transmit the forces to the enamel surface due to their poor flexibility at the debonding process. Therefore, appropriate care must be taken during the debonding brackets [24, 25], requiring different times for different techniques. Sometimes, retaining resin over the dental surface after the debonding processes creates concern as it causes enamel stain in time [26].

The enamel damage and time consumption in the debonding process depend on how the enamel surface was prepared. The class II mesio-occlusal-distal direct resin is more prone to enamel damages. However, lithium disilicate enamel rebuilding gives a good result [27].

The process of bracket removal with inappropriate methods may be durable, damaging, and aching [28]. Hence, research is required to evaluate how different debonding techniques of ceramic brackets require various times.

The current knowledge base for assessing the time-economic debonding technique is still inadequate. Although representing an essential contribution to our knowledge of an effective method for bracket removal, the scientific studies performed do not resolve the problem we face in selecting the patients' best preferred time-economic way of debonding.

Hence, the current research sought to weigh the time required to remove each bracket to propose an optimal debonding technique among the four methods used in the present study.

## 2. Materials and Methods

The current study included 80 left-out premolars of the patient for the orthodontic reason visiting the orthodontic department of Coorg Institute of Dental Sciences under the Rajiv Gandhi University of Health Sciences, Karnataka, Bangalore. Healthy samples without caries, fractures, or broken and structural malformations were considered and preserved in formalin solution. The enamel surface was prepared by polishing the surface with pumice, a siliceous material with a polishing brush. The brackets were debonded using four debonding techniques, i.e., US, DP, LC, and TM. The specimens were divided randomly into four groups with 20 samples, each keeping a 1 : 1 ratio. During debonding, the time taken to debond each bracket was recorded using a stopwatch (ACCUSPLIT Pro Survivor-A601X Stopwatch, clock, extralarge display), and the recorded time was noted for 20 specimens under each group. Afterwards, the data were statistically analyzed.

### 2.1. Statistical Analysis

Descriptive statistics were computed and presented as mean, standard deviation, minimum, and maximum to study the distribution of time required for debonding using each of the four techniques. To compare the difference in mean time needed for the four methods, one-way ANOVA test was applied along with Tukey's HSD for multiple comparisons. Detailed statistical analysis was done using Statistical Package for the Social Sciences (SPSS) software version 22 (IBM Corp., Armonk, New York). A *p* value of less than 0.05 was considered statistically significant. The prior ethical clearance was obtained from the institutional ethics committee of humans (ref no. CIDS/EC/1315).

## 3. Results

The times taken to debond using the four different methods are represented in Figure 1. The time required to debond using the US method ranged from 0.86 to 2.20 seconds, while DP ranged from 0.97 to 2.56 seconds. In the TM, the required debonding time ranged from 0.50 to 2.10 seconds. The least debonding time range was 0.46 to 1.79 seconds required by the LC method.

The mean (±standard deviation) debonding time for the TM was 1.5880 (±0.40339) seconds and was found to be significantly greater among the four debonding techniques used in this study. Debonding with the LC method required the least time with a mean (±standard deviation) value of 0.9880 (±0.31938) seconds. The one-way ANOVA test revealed that the mean times to debond by the four techniques were significantly different (*p* < 0.001), as displayed in Table 1.

Tukey's HSD multiple comparisons revealed that the mean time to debond using the ligature cutter is significantly less than the other three methods (*p* < 0.001).

Simultaneously, there was no significant difference in the mean time to debond between the other three methods compared with one another, as shown in Table 2.

## 4. Discussion

The current study compared different debonding ceramic bracket methods to determine a time-efficient bracket removal technique that agrees with research [2] already done. Though studies are scanty for time evaluation following a debonding approach on ceramic brackets, several studies on the comparison of bracket removal time are available on stainless steel brackets [29–31].

As ceramic brackets' introduction to the orthodontic speciality increases its demand for its esthetic properties [28, 32, 33], this study compares four different ceramic bracket removal methods to find the time-effective plan mentioned in some research studies [11, 20, 34]. The same tasks compared DP, US, and a mixture of both techniques. However, they reported the DP as a more time-consuming technique followed by the US, which contradicts our findings.

The mean time score for the TM of debonding was the highest, followed by the current study's US method, partially supporting a few research outcomes [20, 34].

The mean time of debonding for the TM was significantly greater among the four debonding techniques. In contrast, a review reported the US as a more time-consuming method [35]. Some studies [20, 36, 37] revealed that the debonding time was minimal with the DP method than the US and electrothermal methods, partially agreeing with the current findings. However, the LC method consumed the least time significantly compared to the US, DP, and TM of debonding in the present study. In contrast, studies [20, 36, 37] revealed insignificant differences in the debonding time between the electrothermal and conventional bracket removal methods.

### 4.1. Limitation of the Study

The study sample in the present study was less, and it was an *in vitro* study. Evaluating the relationship of debonding time with the pain induced could have been more interesting, which was not done in this study.

## 5. Conclusion

The ideal less time-consuming bracket removal method is challenging to evaluate as each way responds differently.

Based on the study's outcome, the mean time to debond by the four techniques was found significantly different. The mean time for the TM was considerably greater, followed by the ultrasonic scaler and debonding pliers. Debonding with the LC method requires substantially less time than that of the other three ways. Therefore, as a standard debonding method among the ceramic brackets, the LC technique may be suggested.

## Figures and Tables

**Figure 1:** Time taken to debond by the four different methods. US: ultrasonic scaler; DP: debonding plier; LC: ligature cutter; TN: thermal method.

**Table 1:** Mean time to debond using different debonding methods.

Method used	Mean	*N*	Std. deviation	Minimum	Maximum	*F* for one-way ANOVA (*p* value)
US	1.4605	20	0.27884	0.86	2.20	10.94 (0.001)
DP	1.4260	20	0.39531	0.97	2.56	
LC	0.9880	20	0.31938	0.46	1.79	
TM	1.5880	20	0.40339	0.50	2.10	

US: ultrasonic scaler; DP: debonding plier; LC: ligature cutter; TN: thermal method.

**Table 2:** Tukey's multiple comparison test for the time taken between the four different debonding methods.

Method (I)	Method (J)	Mean difference (I-J)	*p* value	95% confidence interval	
				Lower bound	Upper bound
US	DP	0.03450	0.990	−0.2588	0.3278
	LC	0.47250^*∗*^	0.001	0.1792	0.7658
	TM	−0.12750	0.665	−0.4208	0.1658

DP	US	−0.03450	0.990	−0.3278	0.2588
	LC	0.43800^*∗*^	0.001	0.1447	0.7313
	TM	−0.16200	0.472	−0.4553	0.1313

LC	US	−0.47250^*∗*^	0.001	−0.7658	−0.1792
	DP	−0.43800^*∗*^	0.001	−0.7313	−0.1447
	TM	−0.60000^*∗*^	0.001	−0.8933	−0.3067

TM	US	0.12750	0.665	−0.1658	0.4208
	DP	0.16200	0.472	−0.1313	0.4553
	LC	0.60000^*∗*^	0.001	0.3067	0.8933

US: ultrasonic scaler; DP: debonding plier; LC: ligature cutter; TN: thermal method. ^∗^The mean difference is significant as the *p* value < 0.05.

## Data Availability

The data used to support the findings of this study are included within the article.
